The article "The Effect of Resveratrol on Blood Glucose and Blood Lipids in Rats with Gestational Diabetes Mellitus" was published in 2021. Journal: Evid Based Complement Alternat Med.

# The Effect of Resveratrol on Blood Glucose and Blood Lipids in Rats with Gestational Diabetes Mellitus

**DOI:** 10.1155/2021/2956795

**Published:** 2021-10-19

**Authors:** Guanli Zhang, Xiuli Wang, Baofeng Ren, Qiongqiong Zhao, Fang Zhang

**Affiliations:** ^1^Department of Obstetrics, Yantaishan Hospital, Yantai 264000, Shandong Province, China; ^2^Department of Obstetrics, Chengyang People's Hospital, Qingdao 266000, Shandong Province, China; ^3^Medical Insurance Department, Zhangqiu District People's Hospital, Jinan,250200, Shandong Province, China; ^4^Department of Paediatrics (II), Zhangqiu District People's Hospital, Jinan 250200, Shandong Province, China; ^5^Department of Clinical Laboratory, Jinan Central Hospital, Cheeloo College of Medicine, Shandong University, Jinan 250013, Shandong Province, China

## Abstract

**Background:**

Previous studies have reported that resveratrol has various biological effects such as anti-inflammatory, antioxidant, and antitumor. This study aimed to investigate the effects of resveratrol on blood glucose and blood lipids in rats with gestational diabetes mellitus (GDM).

**Methods:**

The rat diabetes model was prepared by one-time intraperitoneal injection of streptozotocin (STZ, 35 mg/kg). Fasting blood glucose was measured by using a blood glucose meter. The ELISA method was used to detect the levels of insulin, leptin, adiponectin, resistin, TNF-*α*, and IL-6. The content of TC, TG, LDL-C, and HDL-C was determined by using an automatic biochemical detector.

**Results:**

Compared with the GDM group, the insulin level in the resveratrol (120 and 240 mg/kg) treatment group was significantly increased. But, the blood glucose level and body weight were significantly reduced. The content of TC, TG, and LDL-C in the resveratrol (240 mg/kg) treatment group was significantly reduced, and the content of HDL-C was significantly increased. In addition, leptin, resistin, TNF-*α*, and IL-6 levels in the 240 mg/kg resveratrol treatment group were significantly reduced, and adiponectin was significantly increased. Also, resveratrol (240 mg/kg) was stronger than metformin hydrochloride in improving insulin secretion and regulating blood lipids and adipokine content.

**Conclusion:**

Resveratrol has a dose-dependent effect on GDM rats to increase insulin secretion, reduce blood glucose and body weight, and regulate blood lipids and plasma adipokines.

## 1. Introduction

Gestational diabetes mellitus (GDM) refers to diabetes or impaired glucose tolerance that occurs or is first discovered during pregnancy [1]. Although the abnormal glucose metabolism of GDM patients can return to normal after delivery, the chance of developing type 2 diabetes will increase in the future [2]. GDM is extremely harmful to mothers and babies and may cause preeclampsia, premature rupture of membranes, and premature delivery [3]. The incidence of fetal malformations is 3 to 4 times that of the normal control group [4]. Therefore, timely treatment of GDM is of great significance to the health of mothers and infants and can also effectively reduce the incidence of diabetes in the future.

The etiology and pathogenesis of GDM are extremely complex and have not yet been fully elucidated. The main features of glucose metabolism during pregnancy are increased glucose demand, increased insulin resistance, and relatively insufficient insulin secretion [5]. This may cause GDM in some pregnant women. GDM is more common in people who are obese or overweight, people who have a long-term high-sugar and high-fat diet, people who have a family history of diabetes, and elderly pregnant women [6]. Hyperglycemia can cause abnormal embryonic development and even death, and the incidence of miscarriage can reach 15% to 30% [7]. GDM patients are 2 to 4 times more likely to develop high blood pressure during pregnancy than nondiabetic pregnant women. This may be related to the presence of severe insulin resistance and hyperinsulinemia [8]. In addition, it has been found that obesity, lipid metabolism disorders, and abnormal secretion of adipocytokines in adipose tissue play a very critical role in the pathogenesis of GDM [9]. Therefore, it is very important for GDM patients to find drugs that can lower blood glucose and blood lipids and have fewer side effects.

Resveratrol is a kind of polyphenol compounds, mainly derived from peanuts, grapes (red wine), knotweed, mulberries, and other plants [10]. Resveratrol is a natural antioxidant that can reduce blood viscosity. Resveratrol can also inhibit platelet coagulation and vasodilation and maintain blood flow [11]. Resveratrol has an effect on inhibiting atherosclerosis and preventing coronary heart disease, ischemic heart disease, and hyperlipidemia [12]. Because resveratrol has a variety of biological and pharmacological activities, it is widely used in food, medicine, health-care products, and cosmetics [13]. In addition, it has been found that resveratrol can control and reduce the body weight of obese rats [14]. Therefore, we speculate that resveratrol may play a role in reducing blood glucose and blood lipids in patients with GDM.

In this study, a one-time intraperitoneal injection of streptozotocin (STZ) was used to prepare a 5-day GDM rat model. The purpose of this study is to explore the regulating effect of resveratrol on blood glucose and blood lipid levels in GDM rats.

## 2. Materials and Methods

### 2.1. Animals

Female and male SD rats (SPF, 180–220 g) were purchased from the Hebei Experimental Animal Center (Shijiazhuang, China). All rats were reared in the animal room in a suitable breeding environment (temperature 23 ∼ 25°C, relative humidity 65 ∼ 70%). The photoperiod was 12 h: 12 h. The animal experiment was approved by the Experimental Animal Committee of Jinan Central Hospital.

### 2.2. GDM Model

After the female rats were fed a high-fat diet for 8 weeks in the animal room, the estrus cycle was measured by the vaginal smear method. Female rats and male rats in pre-estrus were caged overnight at a ratio of 1 : 2. Next day, the vaginal smear was examined under a microscope, and the sperm observed was determined to be a pregnant mouse. After 5 days of pregnancy, STZ (35 mg/kg, Yi Sheng Biotechnology Co., LTD, Shanghai, China) was injected intraperitoneally to make a GDM model. After 72 h, when the fasting blood glucose stabilized at 13.5 mmol/L, the model was established successfully. 100 GDM rats were randomly divided into 5 groups: the GDM model control group (GDM-NC), resveratrol 60, 120, and 240 mg/kg treatment group, and metformin hydrochloride (200 mg/kg) positive control group. Another 20 SD rats with 5 days gestation were taken as the normal pregnancy control group. Rats in each group were given continuous administration for 2 weeks (1 time/day). The normal pregnancy control group and GDM-NC group were given equal volume of normal saline. After 2 weeks of treatment, the rats in each group were weighed and recorded with an electronic balance.

### 2.3. Blood Glucose and Insulin Level

A blood glucose meter (ACCU-CHEK, Shanghai, China) was used to measure the abdominal blood glucose of each group on the 0th, 7th, and 14th day of treatment. The insulin level in rat plasma was measured with an ELISA kit (MILLIPORE, Beijing, China).

### 2.4. Detection of TC, TG, LDL-C, and HDL-C in Serum

Two weeks after the drug treatment, urethane (Beijing Chemical Reagent Company, Beijing, China) was injected intraperitoneally for anesthesia. Blood was collected from the abdominal aorta, and the upper serum was collected after centrifugation at 2000 rpm for 5 min. An automatic biochemical detector (Wuhan Jingcheng Weiye Medical Instruments Co., Ltd., Wuhan, China) was used to determine the serum levels of TC, TG, LDL-C, and HDL-C in each group.

### 2.5. Detection of Leptin, Adiponectin, Resistin, TNF-*α*, and IL-6 Levels in Plasma

After 2 weeks of treatment, urethane was injected intraperitoneally for anesthesia. Blood was taken from the abdominal aorta and anticoagulated with heparin. An ELISA kit (MILLIPORE, Beijing, China) was used to determine the levels of leptin, adiponectin, resistin, TNF-*α*, and IL-6 in plasma.

### 2.6. Statistical Analysis

All experiments were repeated 3 times. SPSS 22.0 (IBM Corp.) was used for statistical analysis. All experimental data were displayed as mean ± SD. Paired Student's *t* test was used to analyze the parameter comparison between the two groups. *P* < 0.05 was considered to indicate a statistically significant difference.

## 3. Results

### 3.1. The Effects of Resveratrol on Fasting Blood Glucose and Insulin Levels in GDM Rats

Compared with the normal pregnancy control group, the fasting blood glucose level of the GDM-NC group was significantly increased (*P* < 0.01, Table 1). After 2 weeks of treatment with resveratrol (120 and 240 mg/kg) and metformin hydrochloride (200 mg/kg), blood glucose levels were significantly lower than those in the GDM-NC group (*P* < 0.05, Table 1). Compared with the normal pregnancy control group, the insulin level of the GDM-NC group was significantly reduced (*P* < 0.01, Table 2). After 2 weeks of treatment with resveratrol (120 and 240 mg/kg) and metformin (200 mg/kg), insulin levels were significantly increased compared with the GDM-NC group (*P* < 0.05, Table 2). The abovementioned results indicate that resveratrol can increase insulin levels and lower blood glucose in GDM rats.

### 3.2. The Effect of Resveratrol on the Weight of Rats with GDM

Compared with the normal pregnancy control group, the body weight of the GDM-NC group was increased significantly (*P* < 0.01, Figure 1). After 2 weeks of treatment with resveratrol (120 and 240 mg/kg) and metformin hydrochloride (200 mg/kg), the body weight of GDM rats was significantly reduced compared with the GDM-NC group (*P* < 0.05, Figure 1). These results indicate that resveratrol can reduce the body weight of GDM rats.

### 3.3. The Effect of Resveratrol on the Content of TC, TG, LDL-C, and HDL-C in the Serum of GDM Rats

Compared with the normal pregnancy control group, the serum levels of TC, TG, and LDL-C in the GDM-NC group were significantly increased, and the content of HDL-C was significantly decreased (*P* < 0.01, Figures 2(a)–2(d)). After 2 weeks of treatment with resveratrol (120 and 240 mg/kg), serum levels of TC and TG were lower than those in the GDM-NC group (*P* < 0.05, Figures 2(a), 2(b)). Among them, the LDL-C content of the resveratrol (240 mg/kg) treatment group was significantly reduced. Also, the HDL-C content of the resveratrol (240 mg/kg) treatment group was significantly increased (*P* < 0.05, Figures 2(c), 2(d)). Compared with the metformin hydrochloride treatment group, the resveratrol (240 mg/kg) treatment group had a better effect on lowering blood lipids. These results indicate that resveratrol can effectively reduce blood lipid levels in GDM rats.

### 3.4. The Effect of Resveratrol on the Levels of Leptin, Adiponectin, Resistin, TNF-*α*, and IL-6 in the Plasma of Rats with GDM

Compared with the normal pregnancy control group, the plasma levels of leptin, resistin, TNF-*α*, and IL-6 in the GDM-NC group were significantly increased, and the adiponectin level was significantly reduced (*P* < 0.01, Figures 3(a)–3(e)). After 2 weeks of treatment with resveratrol (240 mg/kg), compared with the GDM-NC group, the plasma levels of leptin, resistin, TNF-*α*, and IL-6 in GDM rats were significantly reduced (*P* < 0.05, Figures 3(a), 3(c)–3(e)). In addition, adiponectin was significantly increased in the 240 mg/kg resveratrol treatment group, while resistin was significantly decreased (*P* < 0.05, Figure 3(b)). Compared with the metformin hydrochloride treatment group, the plasma levels of leptin, resistin, TNF-*α*, and IL-6 in the resveratrol (240 mg/kg) treatment group were significantly increased. Also, the adiponectin level was apparently decreased (Figures 3(a)–3(e)). The abovementioned results indicate that resveratrol may reduce blood lipids in GDM rats by regulating these adipocytokines.

## 4. Discussion

GDM is one of the common complications of pregnancy. Hyperglycemia during pregnancy not only endangers the health of the mother but also has an adverse effect on the fetus [15]. At present, the main clinical treatments for GDM are insulin and oral hypoglycemic drugs metformin and thiazolidinedione. However, these drugs have large side effects and easily pass through the placental barrier [16]. Therefore, the development of hypoglycemic drugs suitable for pregnant women has important clinical significance.

Resveratrol is a naturally occurring nonflavonoid polyphenol compound, which is widely present in natural plants such as grape, knotweed, cassia seed, and peanut [17]. Previous studies have reported that resveratrol has various biological effects such as anti-inflammatory, antioxidant, and antitumor [18, 19]. In this study, we found that insulin secretion levels and fasting blood glucose levels in GDM rats were significantly increased after 2 weeks of resveratrol treatment. The levels of TC, TG, and LDL-C in the resveratrol group were significantly reduced, while the level of HDL-C was significantly increased. In addition, the weight of rats in the resveratrol group was significantly reduced. It has been shown that obesity and lipid metabolism disorders are very dangerous predisposing factors for diabetes [20]. Therefore, the hypolipidemic effect of resveratrol is of great significance to the treatment of GDM.

In addition, we also found that the levels of leptin, TNF-*α*, and IL-6 in the plasma of resveratrol GDM rats were significantly reduced. Leptin has been reported to inhibit the secretion of insulin and exert a negative feedback effect between blood insulin and adipose tissue [21]. TNF-*α* and IL-6 can affect the phosphorylation of insulin-sensitive cells, block insulin signal transduction, and cause abnormal glucose metabolism [22]. This study also found that resveratrol can increase adiponectin levels and reduce resistin levels. Resistin can reduce the uptake of glucose by adipose tissue and inhibit the signal transduction pathway of insulin [23]. Adiponectin can reduce the occurrence and development of diabetes by improving insulin sensitivity [24]. These results indicate that resveratrol has a dose-dependent effect on GDM rats to increase insulin secretion, reduce blood glucose, reduce body weight, and regulate blood lipids and plasma adipokines. Moreover, resveratrol was stronger than metformin hydrochloride in improving insulin secretion and regulating blood lipids and adipokines. However, the specific mechanisms of resveratrol for regulating blood sugar and blood lipids are still unclear. This is also the main problem that we need to solve in the future.

## 5. Conclusions

Resveratrol has a dose-dependent effect on reducing blood glucose and blood lipids in GDM rats. Resveratrol can also treat GDM by promoting insulin secretion and regulating adipokines. However, this study has not yet elucidated the specific regulatory mechanism of resveratrol in GDM. Therefore, the regulatory mechanism of resveratrol in GDM will be explored in the future.

## Figures and Tables

**Figure 1:** The effect of resveratrol on the weight of rats with GDM. The body weight of rats with GDM in the resveratrol (60, 120, 240 mg/kg) treatment group and metformin hydrochloride treatment group was compared with that in the GDM-NC group. ^∗^*P* < 0.05, ^∗∗^*P* < 0.01.

**Figure 2:** The effect of resveratrol on the content of TC, TG, LDL-C, and HDL-C in the serum of GDM rats. (a–d) The TC, TG, LDL-C, and HDL-C levels in of rats with GDM in the resveratrol (60, 120, 240 mg/kg) treatment group and metformin hydrochloride treatment group were compared with those in the GDM-NC group. *∗P* < 0.05, *∗∗P* < 0.01.

**Figure 3:** The effect of resveratrol on the levels of leptin, adiponectin, resistin, TNF-*α*, and IL-6 in the plasma of rats with GDM. (a–e) The leptin, adiponectin, resistin, TNF-*α*, and IL-6 levels of rats with GDM in the resveratrol (60, 120, 240 mg/kg) treatment group and metformin hydrochloride treatment group were compared with those in the GDM-NC group. *∗P* < 0.05, *∗∗P* < 0.01.

**Table 1:** The effect of resveratrol on fasting blood glucose level in GDM rats.

Group	Dosage (mg/kg)	0^th^ day (mmol/L)	7^th^ day (mmol/L)	14^th^ day (mmol/L)
Normal pregnancy		6.1 ± 0.7^∗∗^	6.2 ± 0.6^∗∗^	6.3 ± 0.5^∗∗^
GDM-NC		16.3 ± 2.2	16.4 ± 2.3	16.1 ± 2.5
Resveratrol	60	16.6 ± 2.3	15.4 ± 2.1	14.9 ± 2.1
	120	16.3 ± 2.0	13.5 ± 1.8^∗^	12.8 ± 1.8^∗^
	240	16.2 ± 1.8	12.2 ± 1.6^∗^	9.7 ± 1.5^∗∗^

Metformin hydrochloride	200	16.4 ± 2.2	10.9 ± 1.5^∗^	8.8 ± 1.3^∗∗^

Compared with the GDM-NC group, *∗P* < 0.05, *∗∗P* < 0.01.

**Table 2:** The effect of resveratrol on insulin level in GDM rats.

Group	Dosage (mg/kg)	0 day (mmol/L)	7 day (mmol/L)	14 day (mmol/L)
Normal pregnancy		13.2 ± 2.3^∗∗^	13.3 ± 2.1^∗∗^	13.1 ± 2.4^∗∗^
GDM-NC		5.6 ± 1.1	5.5 ± 0.9	5.6 ± 1.0
Resveratrol	60	5.6 ± 1.2	6.8 ± 1.4	7.1 ± 1.5
	120	5.5 ± 0.9	7.6 ± 1.5^∗^	8.5 ± 1.3^∗^
	240	5.4 ± 1.0	10.3 ± 1.6^∗^	12.2 ± 1.2^∗∗^

Metformin hydrochloride	200	5.5 ± 2.2	7.4 ± 1.5^∗^	8.6 ± 1.6^∗^

Compared with the GDM-NC group, ^∗^*P* < 0.05, ^∗∗^*P* < 0.01.

## Data Availability

The datasets used during the present study are available from the corresponding author upon reasonable request.
